# FE-SEM Evaluation of Dental Specimens Prepared by Different Methods for *In Vitro* Contamination

**DOI:** 10.1155/2012/748471

**Published:** 2012-03-11

**Authors:** Vitor Cesar Nakamura, Simony Hidee Hamoy Kataoka, Giulio Gavini, Patrícia Helena Ferrari, Silvana Cai

**Affiliations:** ^1^Department of Dentistry, School of Dentistry, University of São Paulo, São Paulo, SP, Brazil; ^2^Department of Oral Microbiology, Biomedical Science Institute, University of São Paulo, São Paulo, SP, Brazil

## Abstract

*Objective*. To evaluate through FE-SEM the cleanliness and dentinal alterations promoted by different methods of dental sample preparation. *Methods*. Twenty-five human single-rooted teeth were used. The teeth were cleaned and autoclaved in wet medium and randomly divided into 5 groups (*n* = 5), according to the preparation methods employed—control group: no solutions applied; group 1: cement removal and irrigation with 5.25% NaOCl  + 17 % EDTA for 4 minutes each; group 2: 17%  EDTA + 2.5% NaOCl (4 minutes ultrasonic bath); group 3: cement removal and 17%  EDTA + 5.25%  NaOCl + phosphate buffer solution + distilled water (10 minutes ultrasonic); group 4: 17%  EDTA + 5.25% NaOCl (3 minutes ultrasonic bath). Specimens were analyzed by field emission scanning electron microscope (FE-SEM), at 1500x magnification. Data were submitted to qualitative analysis according to a scoring system and submitted to Kruskal-Wallis test. *Results*. In ascending order, as to bind parameters, (i) cleanliness: control, group 2, group 3, group 5, and group 4, (ii) dentinal alterations: group 1, group 5, group 2, group 3, and group 4. *Conclusion*. The proposed protocol was suitable for subsequent microbiological contamination, because it showed less dentinal morphological alterations with increased removal of organic waste.

## 1. Introduction

The presence of microorganisms and their products in the root canal system is the major etiologic agent and plays a fundamental role in the etiology of pulp and periapical diseases [1, 2]. Thus, the microbial control through chemomechanical procedures becomes essential for tissue repair [3]. Due to the complex anatomy of the endodontic space, disinfection should include not only the action of mechanical instruments, but also the use of antimicrobial irrigation solutions, as demonstrated by Bystrom and Sundqvist in 1985 [4]. The use of intracanal medication with antimicrobial profile also shows to be an excellent adjuvant for the decontamination of the endodontic system [5].

In order to test irrigation agents used during the root canal preparation and antibacterial intracanal medications, it is essential to develop laboratorial methods of infection, seeking to simulate, *in vitro*, the situations of infection observed *in vivo*. For this purpose, it is necessary to prepare the human tooth to receive microbial contamination.

According to Haapasalo and Orstavik [6] it is crucial to use 17% EDTA for 4 minutes at 7.7 p.H, and then 5.25% NaOCl, also for 4 minutes, to completely remove the smear layer and increase the dentinal permeability through clearance of the canaliculus, before the experimental contamination by microorganisms. In order to improve microorganisms penetration, these authors proposed the complete removal of the root cementum prior to chemical preparation.

In 1996, Perez and coworkers [7] prepared specimens for further experimental contamination with ultrasonic bath for 4 minutes with 17% EDTA solution followed by 2.5% NaOCl for 4 minutes, to remove the smear layer and any remaining organic tissue.

Vivacqua-Gomes et al. (2005), concerned about the residuals of EDTA and NaOCl inside root canal, proposed an ultrasonic bath with phosphate buffer solution for 10 minutes, after submitting their specimens to ultrasonic baths with 17% EDTA followed by 5.25% NaOCl, for 10 minutes each [5]. To improve microorganism penetration, they also proposed the removal of the cementum layer.

The methods described in previous studies [5–7] are well known and used for microbiological contamination (bacteria and fungi); however it is necessary to evaluate the dentinal morphological alterations when the specimens are subjected to different preparation protocols in order to evaluate which method better imitates conditions observed *in vivo*. Thus, the aim of this study is to evaluate cleanliness and dentinal morphological alterations promoted by different methods of dental sample preparation and compare them with a new proposal.

## 2. Materials and Methods

### 2.1. Selection and Standardization of Teeth

Twenty-five single-rooted human teeth from the human teeth bank of the Faculty of Dentistry (University of São Paulo) were used. They were cleaned and stored in saline solution for a week for hydration. After this procedure, the teeth were autoclaved in wet medium, and their crowns were sectioned with a diamond disk (KG Sorensen, São Paulo, Brazil). Root lengths were standardized to exactly 15 mm and the apical foramen to 0.30 mm with a stainless steel K file, aided by 0.9% saline solution. The experimental groups were divided and treated according to the table below (Table 1).

After the described procedures, all canal entrances and apical foramens were closed with a vegetal sponge in order to prevent dirt to enter and stay attached to the internal canal walls during the split of the roots. The roots were cleaved longitudinally and prepared for FE-SEM analysis.

 Field Emission Scanning Electron Microscope (FE-SEM) is an equipment which works with electrons, instead of light (photons), like conventional Scanning Electron Microscope (SEM). It provides valuable information that is employed to reconstruct a very detailed image of the topography of the surface of the specimen. In addition, the FE-SEM, unlike the conventional SEM, does not require specimen metallization.

 The samples were dehydrated in graded ethanol series (70, 80, 90, and 99%), stored in a dryer for 24 h, and taken to the FE-SEM. Cleanliness and degree of erosion of root canal walls were evaluated at 1.500x magnification. Images were acquired at 3 mm, 6 mm, and 9 mm from the apical vertex of each root. Each image was divided into 16 subareas by overlaying a grid with an image processing software (Adobe Photoshop CS4, Adobe Systems Incorporated, USA).

Blind evaluation was performed by three different observers. Calibration was performed after the examination of 12 specimens jointly. The effectiviness of this calibration (intraexaminer and interexaminer reliability) was verified by means of the Kappa test. Evaluation of the cleanliness of root canal walls was performed using a three-point scoring system [8], as follows: 0 = no smear layer (all tubules clean and visible with no presence of smear layer on the root canal wall surface), 1 = moderate smear layer (visible debris in tubules but no smear layer on the surface of dentin walls), and 2 = heavy smear layer (root canal walls surface and tubules completely covered by smear layer). A similar three-point score system was used to score the degree of erosion of the root canal walls: 0 = no erosion (appearance of peritubular dentin and size of all tubules look normal), 1 = moderate erosion (peritubular dentin was eroded), and 2 = severe erosion (destruction of intertubular dentin, connecting tubules to each other).

## 3. Results

The results were submitted to Kruskal-Wallis test and differences at *P* < 0.05 were considered statically significant (Tables 2 and 3). The computer program used was BioEstat for Windows (version 3.0). 

## 4. Discussion

An endodontic infection differs from another infection due to the fact that endodontic microorganisms are established at nonvascularized areas. This complicates the action of systemic antimicrobial drugs, which are the usual conduct for infection in different organs and tissues. Many researchers have demonstrated the presence of microorganisms all around the dentinal tubules and areas of difficult mechanical access, like isthmus, in teeth with pulpal necrosis associated to apical periodontitis [9, 10]. This way, the reduction of microbial load should be achieved by the local action of instruments in the main canal, associated with chemical substances and intracanal medications [11]. These drugs are used to penetrate into inaccessible sites, contributing, positively, to the repair of the periradicular tissues [12].

Therefore, the goal of recreating *in vitro *infection conditions in the endodontic system is to evaluate different preparation techniques of the radicular canal, associated to different chemicals, as well as to a diversity of drugs of intracanal usage. Human and bovine teeth have been used *in vitro* for such studies [13–15]. However, the preparation of the dental specimens for further contamination is a relevant factor.

Many authors [5–7] have suggested specimen preparation techniques that differ from each other, basically, as for the time and mode of exposition of the radicular canaliculi to substances. The purpose of such approaches is to remove organic remains from pulpal content and inorganic matter resulted from the mechanic standardization of the samples. The standardization consists of a previous mechanical extension of the radicular canal and transversal or longitudinal cuts of the root. As demonstrated in the present study, these alterations on the sample preparation methodology result in significant differences regarding morphological alterations and dirt removal from the dentin circumjacent to the radicular canal. The three methods previously suggested by different authors [5–7] used sodium hypochlorite solutions at 2.5 or 5.25% and the EDTA at 17%: in group 4 PBS and distilled water were also used, and in group 5 just distilled water was added.

 Regarding the cleanliness of the dental walls, groups 3, 4, and 5 showed higher results when compared to groups 1 and 2, which did not differ among each other (Figure 2(a)). On the other hand, groups 4 and 5 showed cleaning scores statistically higher than group 3 (Figure 2(a)). Thus, by analyzing each group, it is noticeable that the methodologies which included ultrasonic bath showed better cleaning results. It can be inferred that these results are consequence of the continuous agitation of the molecules from the solutions used in the radicular canal, when submitted to ultrasound [16]. Furthermore, another factor to be considered is the time of exposition to the substances. None of the analyzed specimens had walls completely free from debris. However, it is relevant to affirm that the groups in which the specimens were exposed to the substances for longer periods under ultrasonic bath had more favorable debris removal scores. These results are in agreement with the ones presented by Kamburis and coworkers [17], who evaluated the relationship between the exposition time to sodium hypochlorite and organic tissue degradation, and with Serper and Calt [18], who demonstrated that longer contact times to EDTA resulted in higher removal of dental magma. 

 As mentioned previously, laboratory research models must reproduce, as accurately as possible, the conditions presented by the host organ, in order to better evaluate the techniques and chemicals employed during the root canal treatment. When considering extracted human teeth, the less morphological alterations to the dentin circumjacent to the root canal during the standardization and preparation of the samples to get contaminated by microorganisms, the greater the similarity to the clinical reality. Therefore, the results for morphological alterations to the dentin when using the method demonstrated by Perez et al. [7] and the methodology proposed by the current study (applied to groups 3 and 5, resp.) showed no statistically significant differences, as well as when each was compared to the results for the control group (group 1). In these three groups the peritubular dentin showed to be complete, with small alterations, suggesting a demineralization process on a few sites. On the other hand, groups 2 and 4 (Figure 2(b)) showed more dentinal alterations when compared to the other groups, particularly in group 4, which had the worst results, and in which images it was possible to observe the presence of generalized demineralization of the dentin, as well as the occurrence of erosions in some sites (Figures 1(j), 1(k), and 1(l)). It is imperative to emphasize that, in both groups 2 and 4, the radicular cement was previously removed [5, 6]. This could have favored a greater flux of substances through the dentinal tubules, from inside the root canal to outside the root, which might have resulted in such differences. Petelin and coworkers [19] demonstrated that the interface between the cement and the radicular dentin forms a barrier which obstructs the liquid diffusion through the dentinal tubules. Undoubtedly, this barrier can enhance the *in vitro* contamination of the dental specimens. However, other studies are necessary to clarify whether the procedure of cement removal could also facilitate the microorganisms' exclusion through chemical ways.

 An indispensable condition to perform reliable studies about agents and instruments to decontaminate the root canal is that the dentinal walls are free from organic remains, smear layer, and dirt and that they have dentinal tubules with openings which favor the penetration of microorganisms. However, the dentin's natural morphological features must be maintained, in order to increase the predictability of the results from these same agents when they are used in clinical situations.

It can be concluded, from the present study, that the new proposal of preparation of the specimens to receive bacterial contamination (methodology applied to group 5) presented favorable results, compared to the other studied methods, for resulting in dentinal walls with little dirt, besides not changing significantly the morphological aspect of the dentin. Nonetheless, the standard analysis of microbial contamination in the different protocols is essential for future studies, in order to resemble the most possible with what occurs *in vivo*.

## Figures and Tables

**Figure 1:** (a–o) FE-SEM images from coronal, middle and apical thirds of samples of each experimental group. Group 1: (a) (coronal), (b) (middle), and (c) (apical) evidence of dirt obscuring the tubules. Group 2: (d) (coronal), (e) (middle), and (f) (apical) dirt were present. In (d) note the absence of dirt, but with morphological alteration. The middle third was clean, however it shows obscured tubules. Group 3: (g) (coronal) destruction of peritubular dentin, (h) (middle) obstruction in some tubules, and (i) (apical) evident dirt obscured in all tubules. Group 4: (j) (coronal), (k) (middle), and (l) (apical) no evidence of dirt in the three thirds, but in all thirds some evidence of intra- and intertubular destruction. Group 5: (m) (coronal), (n) (middle), and (o) (apical) with some bits of dert in the middle third (arrow).

**Figure 2:** (a) Statistical difference between experimental groups by average position of cleanliness scores (B). (b) Statistical difference between experimental groups by average position of morphological alterations scores.

**Table 1:** Treatment applied on control and each experimental group.

Group	N. specimens	Treatment	Reference
1	5	None solution (control group)	—
2	5	5.25% NaOCl + 17% EDTA (pH = 7.7) for 4 minutes each with cement remotion	[6]
3	5	17% EDTA + 2.5% NaOCl for 4 minutes in an ultrasonic bath	[7]
4	5	17% EDTA + 5.25% NaOCl + phosphate buffer solution + distilled water for 10 minutes each in an ultrasonic bath with cement remotion	[5]
5	5	17% EDTA + 5.25% NaOCl + distilled water for 3 minutes in an ultrasonic bath	New proposal

**Table 2:** Mean scores of dirt removal attributed alterations attributed to teeth in groups 1 (control), 2, 3, 4, and 5.

Groups	Scores
1	1.75
2	2.55
3	2.94
4	4.14
5	3.94

**Table 3:** Mean scores of dentinal morphological to teeth in groups 1 (control) 2, 3, 4, and 5.

Groups	Scores
1	2.02
2	2.96
3	2.56
4	3.81
5	1.98
